The article "Effects of Forced Swimming Stress on ERK and Histone H3 Phosphorylation in Limbic Areas of Roman High- and Low-Avoidance Rats" was published in 2017. Journal: PLoS One.

# Effects of Forced Swimming Stress on ERK and Histone H3 Phosphorylation in Limbic Areas of Roman High- and Low-Avoidance Rats

**DOI:** 10.1371/journal.pone.0170093

**Published:** 2017-01-20

**Authors:** Noemi Morello, Ornella Plicato, Maria Antonietta Piludu, Laura Poddighe, Maria Pina Serra, Marina Quartu, Maria Giuseppa Corda, Osvaldo Giorgi, Maurizio Giustetto

**Affiliations:** 1 Department of Neuroscience, University of Turin, Turin, Italy; 2 Department of Life and Environmental Sciences, University of Cagliari, Cagliari, Italy; 3 Department of Biomedical Sciences, University of Cagliari, Monserrato (CA), Italy; 4 National Institute of Neuroscience-Italy, Turin, Italy; Brock University, CANADA

## Abstract

Stressful events evoke molecular adaptations of neural circuits through chromatin remodeling and regulation of gene expression. However, the identity of the molecular pathways activated by stress in experimental models of depression is not fully understood. We investigated the effect of acute forced swimming (FS) on the phosphorylation of the extracellular signal-regulated kinase (ERK)1/2 (pERK) and histone H3 (pH3) in limbic brain areas of genetic models of vulnerability (RLA, Roman low-avoidance rats) and resistance (RHA, Roman high-avoidance rats) to stress-induced depression-like behavior. We demonstrate that FS markedly increased the density of pERK-positive neurons in the infralimbic (ILCx) and the prelimbic area (PrLCx) of the prefrontal cortex (PFCx), the nucleus accumbens, and the dorsal blade of the hippocampal dentate gyrus to the same extent in RLA and RHA rats. In addition, FS induced a significant increase in the intensity of pERK immunoreactivity (IR) in neurons of the PFCx in both rat lines. However, RHA rats showed stronger pERK-IR than RLA rats in the ILCx both under basal and stressed conditions. Moreover, the density of pH3-positive neurons was equally increased by FS in the PFCx of both rat lines. Interestingly, pH3-IR was higher in RHA than RLA rats in PrLCx and ILCx, either under basal conditions or upon FS. Finally, colocalization analysis showed that in the PFCx of both rat lines, almost all pERK-positive cells express pH3, whereas only 50% of the pH3-positive neurons is also pERK-positive. Moreover, FS increased the percentage of neurons that express exclusively pH3, but reduced the percentage of cells expressing exclusively pERK. These results suggest that (i) the distinctive patterns of FS-induced ERK and H3 phosphorylation in the PFCx of RHA and RLA rats may represent molecular signatures of the behavioural traits that distinguish the two lines and (ii) FS-induced H3 phosphorylation is, at least in part, ERK-independent.

## Introduction

The extracellular signal-regulated kinase (ERK) 1/2 is a member of the mitogen-activated protein kinase (MAPK) intracellular signaling cascade that is highly expressed throughout the brain in mature, postmitotic neurons [1]. Phosphorylation activates ERK 1/2 and triggers a signaling cascade involved in multiple cellular processes, such as neuronal growth and proliferation, differentiation, apoptosis and synaptic plasticity, all of which play an essential role in learning and memory [2]. Furthermore, the ERK pathway is activated by a large variety of stressors and is critically involved in the adaptive behavioral responses to acute and chronic stressful stimuli [3–5].

In addition to cytoplasmic substrates (e.g., protein kinases, ion channels, cytoskeletal and synaptic vesicle trafficking proteins), ERK 1/2 can directly or indirectly modify transcription factors and histones [2,6]. These processes lead in turn to the encoding of environmental stimuli by a rapid and long-term regulation of immediate early genes (IEGs), a mechanism that plays a key role in the adaptive responses to stressors, addictive drugs and their associated learning processes [2,5].

Different types of stressors, such as experimental paradigms of acute and chronic stress, can induce specific epigenetic modifications, depending also on the brain region analyzed. Thus, it has been shown that the phosphorylation at Ser 10 of the histone H3 in mature granule neurons of the dentate gyrus (DG) in the hippocampus is increased, in a glucocorticoid-dependent manner, by a psychological acute stress like forced swimming (FS), but is not affected by physical acute or chronic stress (i.e., ether exposure and repeated cold exposure, respectively) [7]. It has also been shown that the concurrent NMDA receptor signaling pathway is involved in the phosphoacetylation of histone H3 in the DG after FS, through the activation of the ERK 1/2 pathway [3,8]. Importantly, such histone H3 modification induces IEGs expression (e.g.: *c-fos* and Egr-1), thereby leading to the consolidation of memories for adaptive responses such as increased immobility in the FS test [3,8,9]. Also in the medial prefrontal cortex (PFCx), an area critically involved in depression and the responses to stressors, acute FS (15 min session) increases ERK 1/2 phosphorylation [10]. To date, however, very little is known about the impact of a psychological acute stress on the epigenetic modifications in this cortical area. In addition, it is unclear whether such epigenetic mechanisms are differentially regulated in genetic animal models showing divergent responses to stress and vulnerability to depression. One of these models is represented by the Roman high-avoidance (RHA) and low-avoidance (RLA) rats, two outbred lines psychogenetically selected from a Wistar stock for respectively rapid *vs*. extremely poor acquisition of active avoidance in a shuttle-box [11–14]. This psychogenetic selection has generated two phenotypes that differ markedly in the behavioral responses to stressors: when exposed to aversive stimuli, RHA rats display a proactive coping style characterized by robust exploratory and motor behaviors, associated with low intensity hypothalamus-pituitary-adrenal (HPA) axis responses, while RLA rats show a reactive coping style consisting of fear-related behaviors like freezing and self-grooming, and elevated HPA axis reactivity [15–17]. Accordingly, RLA rats display less escape-directed behaviors and more immobility in the forced swim test, whereas RHA rats show robust active behaviors such as swimming and climbing. Interestingly, the depression-like behavior of RLA rats in the above test is normalized by subacute and chronic treatment with antidepressant drugs [18,19].

The Roman lines also display differential neurochemical responses to stressors. Brain microdialysis experiments showed that tail-pinch stress and anxiogenic drugs increase the extracellular concentrations of dopamine in the PFCx of RHA, but not RLA rats [20]. It is noteworthy in this context that acute cocaine and other addictive drugs evoke a more pronounced release of dopamine in the PFCx and the nucleus accumbens shell (AcbSh) of RHA *vs*. RLA rats [14,21]. This effect of cocaine is associated with a significant increment in the expression of pERK 1/2 in the infralimbic compartment (ILCx) of the PFCx and the AcbSh of RHA, but not RLA rats [22].

Although the behavioral and neurochemical responses of RHA and RLA rats to a variety of stressors have been well characterized, it is presently unknown whether signaling pathways and epigenetic modifications play a role in their distinct behavioral responses to stress. The present study was, therefore, designed to evaluate the molecular changes evoked by acute stress in the brain of RHA and RLA rats. To this aim, we used immunohistochemistry to investigate the effects of acute FS on the expression of the phosphorylated forms of ERK 1/2 and histone H3 in several limbic areas of both Roman lines.

## Materials and Methods

### Animals

Outbred Roman high- (RHA) and low-avoidance (RLA) male rats from the colony established in 1998 at the University of Cagliari, Italy, were used throughout. Animals were housed in groups of 4 per cage and maintained in a temperature- and humidity-controlled environment (23 ± 1°C and 60 ± 10%, respectively) under a 12 h light-dark cycle (lights on at 8:00 a.m.). Water and standard laboratory food were available *ad libitum*. To minimize stress to the experimental animals, all the maintenance activities in the animal house were carried out by a single attendant. Rats were 3–4 month old at the time of behavioral testing (body weight 350–450 g). All the experiments were conducted in accordance with the European Communities Council Directive 2010/63/EU and approved by the Italian Ministry of Health, by the Bioethical Committee of the University of Turin and by the Ethical Committee for Animal Care and Use of the University of Cagliari. The protocol was approved by the Committee on the Ethics of Animal Experiments of the Italian Ministry of Health (Permit Number: 684/2015 PR). Every possible effort was made to minimize animal pain and discomfort and to reduce the number of experimental subjects.

### Forced swimming

Twelve rats from each line were randomly assigned to one of the following groups: RHA control, i.e., basal (Bs), RHA test, i.e., forced swimming (FS), RLA Bs, and RLA FS (n = 6 for each group). The forced swimming procedure was as described in [18], except for the duration of the swim session. Briefly, 15 min swim sessions were conducted by placing the rats in individual plastic cylinders 58 cm tall and 32 cm in diameter, which were filled with water at 24–25°C to a 40 cm depth to ensure that the animals could not touch the bottom of the cylinder with their tails or hind paws. Control rats (Bs) were left undisturbed in their home cages before anesthesia.

### Immunohistochemistry

At the conclusion of the forced swimming session, animals were deeply anesthetized with an intraperitoneal (i.p.) injection of chloral hydrate (Carlo Erba, Milan, Italy) at the dose of 550 mg/kg/2ml, and transcardially perfused with physiological saline solution (NaCl 0.9% w/v, pH 7.4) followed by 4% paraformaldehyde (PFA) in 0.1 M phosphate buffer (PB). After perfusion, brains were removed and post-fixed overnight in 4% PFA. The brains were then washed in PB and cryoprotected by immersion in 10%, 20%, and 30% sucrose solutions. Coronal sections (30 μm) were cut with a cryostat and stored at -20°C in a solution containing 30% ethylene glycol and 25% glycerol in 0.1 M PB (pH 7.2) until processing. Immunohistochemistry was carried out according to a protocol for free-floating sections. Immunoreactions were performed in at least three cryosections of the regions of interest obtained from each brain. The sections were selected between the following AP coordinates from Bregma, using the rat brain atlas of Paxinos & Watson (1986) as a reference: prefrontal cortex (PFCx), +3.20 mm to +2.70 mm, nucleus accumbens (Acb), +1.00 mm to +0.70 mm, and dentate gyrus (DG), -2.56 mm to -2.80 mm. After being rinsed in PBS (3 x 10 min), sections were immersed in 1% H_2_O_2_ in PBS for 30 min to block endogenous peroxidase activity. After a blocking step in a PBS solution containing 0.5% Triton X-100 and 10% normal goat serum (NGS), sections were incubated overnight at room temperature with one of the following primary antibodies diluted in PBS with 3% normal goat serum (NGS) and 0.05% Triton X-100: (i) mouse monoclonal anti-phospho-ERK (ERK 1/2, T183-Y185; 1:500, Sigma, St. Louis, MO), or (ii) rabbit polyclonal anti-phospho-H3 (Ser10; 1:500, Upstate/Millipore Billerica, MA). On the following day, after 3 rinses in PBS, sections were incubated for 1h with the appropriate biotinylated secondary antibodies (1:250; Vector Labs; Burlingame, CA) diluted in PBS with 3% NGS and 0.05% Triton X-100, followed by 1h incubation in a solution containing a biotin-avidin complex (1:100, Vector Labs). Finally, sections were immersed in a solution containing 3,3’-diaminobenzidine (0.05% DAB in TRIS-HCl, pH 7.6) with 0.01% H_2_O_2_ for 3–4 min, as in [4].

For immunofluorescence experiments, following 3 rinses in PBS and a blocking step in a PBS solution containing 0.5% Triton X-100 and 10% normal donkey serum (NDS), sections were incubated with the primary antibodies. On the following day, after 3 rinses in PBS, sections were immersed for 1h at room temperature in secondary fluorescent antibodies: donkey anti-mouse Alexa Fluor 488 and donkey anti-rabbit Cy3 (1:1000, Jackson ImmunoResearch, West Grove, PA).

After several PBS rinses, the sections were mounted on glass slides and observed with a bright-field microscope (Eclipse 800, Nikon, Japan) equipped with a CCD camera (Axiocam HRc, Zeiss, Germany) or with a confocal microscope (Zeiss LSM-5 Pascal, Germany) for immunofluorescent samples.

### Quantitative analysis of immunohistochemical signals

All the image acquisitions and analyses were conducted by operators that were blind to animal line and treatment. For immunoperoxidase experiments, we used a 10x objective (area 860x680 μm) to collect micrographs from the regions of interest in 3 coronal cryosections for each animal. Anatomical boundaries of selected brain areas were defined according to the rat brain atlas of Paxinos & Watson (1986). The prelimbic (PrLCx) and infralimbic areas (ILCx) of the PFCx were reconstructed acquiring 2–3 overlapping micrographs from both hemispheres using the Photomerge tool in the Photoshop software package (Adobe Systems, San Jose, CA). For immunofluorescence, micrographs from the PrLCx and the ILCx were acquired with a laser scanning confocal microscope (Pinhole: 1.0 Airy unit). Single stack images were acquired using a 40x objective (512 x 512 pixels; pixel size 0.45 x 0.45 μm).

The expression analysis of both pERK and pH3 in the PFCx was restricted to the upper layers due to their activation pattern in this area. One micrograph of the DG of the hippocampus was collected from each section, and the dorsal (Db) and ventral blade (Vb) of the DG as well as the core (AcbCo) and shell (AcbSh) compartments of the Acb were separately analyzed.

The mean density values of immunolabeled cells was calculated manually (n = 5–6 rats for each group) using a public-domain dedicated software (ImageJ, NIH, USA) as described in [4]. The mean immunoreactivity (IR) intensity of either pERK- or pH3-positive cells was measured in a selected area of the PrLCx and the ILCx (area 245 x 400 μm) using a semi-automatic system in ImageJ. Briefly, the free hand tool was used to manually draw boundaries around stained cells and the integrated density was automatically measured; the background intensity (i.e., the integrated signal intensity of a sample area surrounding labeled cells) was determined and subtracted from the signal intensity of each cell in the same region. The mean intensity of the cells measured in each image was calculated and used to determine, firstly, the mean signal intensity of each rat (n = 6 images for each rat) and, secondly, the mean intensity of each experimental group (n = 6 rats for each group). The frequency distribution of IR intensities was analyzed using a 10 bins count whose range was set between the minimum/maximum values detected for each group comparison. For each bin, the number of cells were averaged among rats of each experimental group and their distribution was evaluated. Given the differences in both minimum and maximum intensity values between the test and control groups, they were statistically evaluated separately. Digital images were cropped or merged using Adobe Photoshop (Adobe Systems, San Jose, CA)

### Colocalization analysis

Double fluorescence micrographs from the PrLCx and the ILCx of each experimental group (n = 3 rats) were acquired with a laser scanning confocal microscope using the multi-track mode to avoid fluorescence cross-talk (Pinhole: 1.0 Airy unit). Z-series stacks of 4 consecutive confocal sections spaced by 3 μm were acquired using a 20x objective (1024 x 1024 pixels; pixel size 0.45 x 0.45 μm). The colocalization analysis was performed manually using ImageJ software.

### Statistical analysis

The density of immunostained cells/area in the PrLCx, the ILCx, the AcbSh, and the AcbCo or cells/length in the DG are expressed as the mean ± SEM. Intensity analysis data are indicated as the mean ± SEM value or as frequency distribution. Data were evaluated using the two-way analysis of variance (ANOVA); main factors: rat line (line) and forced swim (FS). When appropriate (i.e., p < 0.05 for the ANOVA main factors or their interaction), pair-wise comparisons were carried out with Bonferroni *post hoc* tests or with the Student’s t-test for independent samples, as indicated in the figure legends. The frequency distribution of signal intensity histograms was evaluated with the χ^2^ test. All the statistical analyses were performed using GraphPad Prism software (La Jolla, CA, USA), with significance set at p < 0.05.

## Results

### Forced swimming increases the density of pERK-expressing neurons in the prefrontal cortex

To investigate the effects of stress on pERK expression in the Roman lines, we probed brain sections, obtained from RHA and RLA rats under baseline conditions (Bs) or submitted to 15 min of FS, with an antibody against the phosphorylated form of ERK 1/2. We initially focused our analysis on the PFCx in view of our previous finding that mild stressors induce a significant increase in dopamine release in the PFCx of RHA, but not RLA rats [20]. For the image analysis we considered two subregions in the PFCx: PrLCx and ILCx, which are distinguishable on the basis of their distinct afferent and efferent connections [23,24] (Fig 1A). As shown in Fig 1B and 1D, FS produced robust ERK activation in the somata and dendritic processes of pyramidal neurons of the upper layers in both RHA and RLA rats. A two-way ANOVA analysis revealed a significant increment in the density of pERK-positive cells after FS in the PFCx of both rat lines (fold-increase *vs*. the respective basal value: PrLCx, RHA 3.3, RLA 3.5; ILCx, RHA 3.6, RLA 3.5; Fig 1C and 1E). However, *post hoc* pair-wise contrasts with the Bonferroni test showed no significant differences between treatment-matched rat lines either in the PrLCx or the ILCx. On the other hand, when the density of pERK-immunostained neurons was expressed as a percentage of the respective normalized basal value, the increment in the expression of pERK elicited by FS in the ILCx was significantly larger in RHA (264 ± 18%) than RLA rats (146 ± 46%) (Student’s t-test for independent samples: p < 0.05, not shown).

**Fig 1:** Effect of FS on pERK-immunostaining in the PrLCx and ILCx of RHA and RLA rats. (**A**) The red boxes denote the PFCx areas where immunohistochemical analyses were performed (Paxinos & Watson; 1986). (**B, D**) Representative micrographs oriented as in (**A**) showing pERK immunostaining in PrLCx (**B**) and ILCx (**D**). (**C, E**) Quantitative analysis of pERK immunolabeled cell density in PrLCx (**C**) and ILCx (**E**). PrLCx: RHA Bs = 26.9 ± 16.7; RLA Bs = 25.0 ± 10.6; RHA FS = 89.5 ± 7.3; RLA FS = 86.9 ± 16.3; two-way ANOVA: (line) F_(1,17)_ = 0.03, n.s.; (FS) F_(1,17)_ = 22.43, p = 0.0002***; (line x FS interaction) F_(1,17)_ = 0.01, n.s.; ILCx: RHA Bs = 35.8 ± 15.8; RLA Bs = 40.1 ± 16.8; RHA FS = 130.3 ± 6.4; RLA FS = 98.7 ± 18,6; two-way ANOVA: (line) F_(1,17)_ = 0.78, n.s.; (FS) F_(1,17)_ = 24.56, p = 0.0001***; (line x FS interaction) F_(1,17)_ = 1.35, n.s. Number of animals in each experimental group: RHA Bs, n = 5; RLA Bs, n = 6; RHA FS, n = 5; RLA FS, n = 5. Scale bar = 50 μm.

### The density of pERK-positive neurons in the nucleus accumbens and dentate gyrus is increased after forced swimming

We then focused our attention on two other brain regions implicated in the adaptive responses to stressors: the Acb and the DG. The Acb plays a pivotal role in stress response processing by integrating neural inputs from the hippocampus, the PFCx and other limbic areas [25]. For image analysis, we considered two anatomically and functionally different compartments of the Acb (Fig 2A): AcbCo and AcbSh ([16] and references therein). As illustrated in Fig 2B and 2D, the number of pERK-positive cells was increased after FS in the two subregions of the Acb in both rat lines and this qualitative observation was confirmed by two-way ANOVA analyses (fold-increase *vs*. the respective basal value: AcbCo, RHA 5.5; RLA 4.6; AcbSh, RHA 5.4; RLA 4.5; Fig 2C and 2E). However, *post hoc* comparisons showed no significant differences in pERK expression across treatment-matched rat lines.

**Fig 2:** Effect of FS on pERK-immunostaining in the Acb. (**A**) The red boxes denote the brain regions where the analyses were performed. The Core (AcbCo) and Shell (AcbSh) subregions were analized separately. (**B**, **D**) Representative micrographs of pERK immunohistochemical labeling in the AcbCo (**B**) and AcbSh (**D**) oriented as in (**A**). (**C**, **E**) Quantitative analysis of pERK immunostained cell density in AcbCo (**C**) and AcbSh (**E**). AcbCo: RHA Bs = 16.9 ± 3.8; RLA Bs = 17.1 ± 0.4; RHA FS = 94.0 ± 20.1; RLA FS = 78.0 ± 12.9; two-way ANOVA: (line) F_(1,18)_ = 0.42, n.s.; (FS): F_(1,18)_ = 32.18, p < 0.0001***; (line x FS interaction) F_(1,18)_ = 0.44, n.s.; Acbsh: RHA Bs = 36.3 ± 12.8; RLA Bs = 42.4 ± 14.8; RHA FS = 193.2 ± 29.1; RLA FS = 188.1 ± 9,7; two-way ANOVA: (line) F_(1,18)_ = 0.00, n.s.; (FS): F_(1,18)_ = 66.07, p < 0.0001***; (line x FS interaction) F_(1,18)_ = 0.09, n.s. Number of animals in each experimental group: RHA Bs, n = 6; RLA Bs, n = 6; RHA FS, n = 5; RLA FS, n = 5. Scale bar = 50 μm.

Recent reports disclosed that the activation of ERK in the DG plays a key role in the retention of memories of stressful events [26,27]. Interestingly, the Db and Vb of the DG show different responsivity to stressors [8], in keeping with the marked differences in the neuroanatomical organization and connectivity of these areas [28]. The analysis of the effects of FS on the expression of pERK 1/2 in DG (Fig 3A), revealed an increase in the number of pERK immunoreactive neurons in the Db of the DG indistinguishable between rat lines, while the Vb subregion was unaffected (Fig 3B). Two-way ANOVA comparison of data confirmed that FS elicited a significant increase in the density of pERK-positive cells in the Db (percent increment over the respective basal value: RHA +150%, RLA +200%) but not in the Vb of either rat line (Fig 3C and 3D). On the other hand, no differences in pERK expression were found across treatment-matched rat lines.

**Fig 3:** Effect of FS on pERK-immunostaining in the DG. (**A**) The red box indicates the brain region where the analysis was performed. The DG was further divided into dorsal (Db) and ventral (Vb) blades. (**B**) Representative micrographs of Db and Vb of the DG oriented as in (**A**). (**C**, **D**) Quantitative analysis of pERK immunostained cell density in the Db (**C**) and Vb (**D**) of the DG. Db: RHA Bs = 3.75 ± 1.09; RLA Bs = 3.02 ± 0.39; RHA FS = 9.69 ± 1.23; RLA FS = 9.37 ± 1.01; two-way ANOVA: (line) F_(1,19)_ = 0.28, n.s.; (FS) F_(1,19)_ = 37.16, p < 0.0001***; (line x FS interaction) F_(1,19)_ = 0.04, n.s.; Vb: RHA Bs = 3.08 ± 0.68; RLA Bs = 2.83 ± 0.57; RHA FS = 4.72 ± 0.62; RLA FS = 3.50 ± 0.38; two-way ANOVA (line) F_(1,19)_ = 1.54, n.s.; (FS): F_(1,19)_ = 3.77, p = 0.06; (line x FS interaction) F_(1,19)_ = 0.66, n.s.). Number of animals in each experimental group: RHA Bs, n = 6; RLA Bs, n = 6; RHA FS, n = 5; RLA FS, n = 5. Scale bar = 50 μm.

### The intensity of pERK immunolabelling differs between RHA and RLA rats both under basal and stressful conditions

To investigate the effects of FS on the cellular activation of ERK, we also analyzed the immunosignal intensity of pERK in neurons of the PFCx of both lines (Fig 4A). We performed this measurement based on the assumption that the intensity of cellular labeling is directly proportional to the level of ERK activation. As shown in Fig 4B and 4C, FS significantly increased mean staining intensity for pERK in the somata of neurons of the ILCx in both RHA and RLA rats (percent increase over the respective basal value: RHA, 46%; RLA, 23%), but not in the PrLCx of either line, although a tendency toward a statistically significant increase of pERK intensity was observed in the PrLCx of RHA rats after FS (RHA Bs *vs*. RHA FS Student’s t-test for independent samples: p = 0.08). On the other hand, *post hoc* contrasts showed no significant differences across lines in both frontocortical subregions, either under basal conditions or after FS.

**Fig 4:** Effect of FS on the intensity of pERK expression in PFCx: peroxidase immunolabelling. (**A**) Representative micrographs showing pERK immunostaining in pyramidal neurons of the upper layers of the ILCx of RLA animals under basal condition and after FS. Arrowheads indicate pERK-expressing neurons with different level of intensity: black arrowhead at higher intensity and white arrowhead at lower intensity. (**B**, **C**) Quantitative analysis of pERK-labeling intensity in the PrLCx (**B**) and the ILCx (**C**). PrLCx: RHA Bs = 0.11 ± 0.02; RLA Bs = 0.10 ± 0.02; RHA FS = 0.16 ± 0.01; RLA FS = 0.12 ± 0.01; two-way ANOVA: (line) F_(1,18)_ = 1.50, n.s.; (FS): F_(1,18)_ = 3.74, p = 0.06; (line x FS interaction) F_(1,18)_ = 1.45, n.s.); ILCx: RHA Bs = 0.13 ± 0.02; RLA Bs = 0.13 ± 0.02; RHA FS = 0.19 ± 0.02; RLA FS = 0,16 ± 0,02; two-way ANOVA: (line) F_(1,18)_ = 0.51, n.s.; (FS): F_(1,18)_ = 5.65, p = 0.03*; (line x FS interaction) F_(1,18)_ = 0.32, n.s. Number of animals in each experimental group: RHA Bs, n = 6; RLA Bs, n = 6; RHA FS, n = 5; RLA FS, n = 5. Scale bar = 20 μm.

The pERK IR had a very narrow values range in our immunoperoxidase experiments and almost reached signal saturation in most cells. Therefore, to further analyze variations in pERK expression in the PFCx we turned to immunofluorescence and confocal microscopy. Notably, two-way ANOVA analysis revealed that RHA rats show higher pERK immunostaining intensity than RLA rats in the ILCx but not in the PrLCx (two-way ANOVA (line) in Fig 5B and 5C). At variance with the DAB staining results (Fig 4C), we found that FS significantly increased, at the same extent, pERK immunofluorescence in both ILCx and PrLCx of both Roman lines (fold-increase *vs*. the respective basal value: PrLCx, RHA 1.5; RLA 1.4; ILCx, RHA 1.4, RLA 1.5; two-way ANOVA (FS) in Fig 5B and 5C). Interestingly, the frequency distribution analysis of the pERK immunofluorescence signal (Fig 5D–5G) revealed that RHA rats show a significantly larger number of high-intensity labeled cells than RLA animals in the ILCx both under basal and stressed conditions. Altogether, these data indicate that the phosphorylation of ERK in the PFCx is regulated by FS and that RHA rats show increased levels of pERK compared to RLA rats.

**Fig 5:** Effect of FS on the intensity of pERK expression in PFCx: immunofluorescence labelling. (**A**) Representative high magnification images showing pERK immunofluorescence in ILCx of RLA animals under basal condition and after FS. Arrowheads indicate pERK-expressing neurons with different levels of immunostaining intensity (solid arrowhead: higher intensity; open arrowhead: lower intensity). (**B**, **C**) Quantitative analysis of pERK-labeling intensity in PrLCx (**B**) and ILCx (**C**). PrLCx: RHA Bs = 52.29 ± 1.79; RLA Bs = 50.71 ± 1.91; RHA FS = 76.79 ± 1.57; RLA FS = 71.05 ± 4.18; two-way ANOVA: (line) F_(1,16)_ = 2.00, n.s.; (FS) F_(1,16)_ = 75.05, p < 0.0001***; (line x FS interaction) F_(1,16)_ = 0.65, n.s.; ILCx: RHA Bs = 63.41 ± 4.58; RLA Bs = 54.76 ± 3.65; RHA FS = 88.17 ± 1.60; RLA FS = 80.75 ± 4.03; two-way ANOVA: (line) F_(1,16)_ = 4.85, p = 0.043^$^; (FS): F_(1,16)_ = 48.41, p < 0.0001***; (line x FS interaction) F_(1,16)_ = 0.03, n.s. (**D-G**) Quantitative analysis of pERK-labeling intensity distributions in the PrLCx (**D**, **E**) and the ILCx (**F**, **G**) of each experimental group. PrLCx χ^2^ test: RHA Bs *vs* RLA Bs, n.s.; RHA FS *vs* RLA FS, n.s.; ILCx χ^2^ test: RHA Bs > RLA Bs, p < 0.001^###^; RHA FS > RLA FS, p < 0.01^##^). Number of animals in each experimental group: RHA Bs, n = 5; RLA Bs, n = 5; RHA FS, n = 5; RLA FS, n = 5. Scale bar = 50 μm.

### Forced swimming increases histone H3 phosphorylation in the PrLCx and ILCx

Stress-induced ERK 1/2 phosphorylation may produce an increase in the phospho-acetylation of histone H3, which is followed by the transcription of genes involved in the retention of the stressful event [2]. We therefore examined the effect of FS on the expression of pH3 in the PFCx, an area where we detected an increase in ERK activation in both Roman lines upon FS. Because antibodies against the acetylated forms of H3 yield an elevated immunohistochemical signal already at basal conditions, thus making more likely to underestimate changes induced by FS [4] we probed PFCx sections from RHA and RLA rats with an antibody against the phosphorylated form (Ser10) of H3. As shown in Fig 6, the density of pH3-positive cells in the PrLCx and ILCx was relatively low at basal state while FS produced a sharp increase of labeled neurons in both rat lines (Fig 6A and 6B). Two-way ANOVA analyses confirmed that FS induced an increment in the density of pH3-positive cells in the PrLCx of both RHA and RLA rats (fold-increase *vs*. the respective basal value: RHA 2.6, RLA 2.6, Fig 6C). Likewise, in the ILCx, FS induced a marked increment in the number of pH3-positive cells in both lines (fold-increase *vs*. the respective basal value: RHA 2.1, RLA 2.1. Fig 6D). However, *post hoc* contrasts showed no significant differences across rat lines, either under basal conditions or after FS. To the best of our knowledge, this is the first report showing that FS-induced stress strongly activates the phosphorylation of H3 in the rat PFCx.

**Fig 6:** FS increases the phosphorylation of histone H3 in the PrLCx and ILCx of RLA and RHA rat lines. (**A** and **B**) Representative micrographs showing pH3 immunohistochemical labeling in the PrLCx (**A**) and the ILCx (**B**) of each experimental group. (**C**, **D**) Quantitative analysis of pH3 labeled cell density in PrLCx (**C**) and ILCx (**D**). PrLCx: RHA Bs = 109.8 ± 28.1; RLA Bs = 127.5 ± 13.4; RHA FS = 288.8 ± 44.6; RLA FS = 338.6 ± 30.7; two-way ANOVA: (line) F_(1,18)_ = 1.17, n.s.; (FS) F_(1,18)_ = 39.01, p < 0.0001***; (line x FS interaction) F_(1,18)_ = 0.26, n.s.; ILCx: RHA Bs = 97.4 ± 23.7; RLA Bs = 100.8 ± 16.6; RHA FS = 202.1 ± 18.9; RLA FS = 214.0 ± 9.9; two-way ANOVA: (line) F_(1,18)_ = 0.16, n.s.; (FS) F_(1,18)_ = 32.76, p < 0.0001***; (line x FS interaction) F_(1,18)_ = 0.05, n.s. Number of animals in each experimental group: RHA Bs, n = 6; RLA Bs, n = 6; RHA FS, n = 6; RLA FS, n = 5. Scale bar = 50 μm.

### The intensity of pH3 immunolabeling in the PFCx is regulated differently by forced swimming in RHA *vs*. RLA rats

Because pH3 immunoreactivity in the PFCx showed a wide range of intensities (Fig 6A and 6B), we evaluated the intensity of the neuronal pH3 immunolabeling (Fig 7A) across rat lines and conditions. Interestingly, the two-way ANOVA analysis revealed differences between the two rat lines with RHA showing higher pH3 immunostaining intensity than RLA rats (two-way ANOVA (line) in Fig 7B and 7C). Thus, under basal conditions (Fig 7B and 7C) we found that in the PrLCx the mean pH3 signal intensity did not differ significantly across lines (RHA Bs, 0.06 ± 0.004; RLA Bs, 0.06 ± 0.004; Student’s t-test for independent samples: n.s.), whereas it was higher in RHA *vs*. RLA rats in the ILCx (RHA Bs, 0.07 ± 0.003, RLA Bs, 0.05 ± 0.003; Student’s t-test for independent samples: p < 0.05). Moreover, the frequency distribution analysis of pH3 staining intensity under basal conditions revealed a significantly larger number of high-intensity labeled cells in RHA *vs*. RLA rats in both areas of the PFCx (Fig 7D and 7F). In addition, FS significantly increased pH3 immunostaining intensity in the PrLCx and ILCx of both Roman lines (fold-increase *vs*. the respective basal value: PrLCx, RHA 2.0; RLA 1.7; ILCx, RHA 1.9, RLA 1.8, Fig 7B and 7C). Notably, we found significant differences in pH3 immunostaining intensity across lines after FS in both frontocortical subregions (two-way ANOVA (FS); Bonferroni post-hoc contrasts: p < 0.05) with the RHA line showing higher mean intensity values than the RLA line. In keeping with these results, the frequency distribution analysis of pH3 staining intensity (Fig 7E and 7G) revealed a significantly larger number of high-intensity labeled cells in RHA *vs*. RLA rats in both the PrLCx and the ILCx. These results suggest that experience-dependent epigenetic changes of histone H3 are differentially regulated in RHA *vs*. RLA rats.

**Fig 7:** Differential effects of FS on the intensity of pH3 immunostaining in the PrLCx and the ILCx. (**A**) Representative high magnification images showing pH3 immunostaining in ILCx of RLA animals under basal conditions and after FS. Arrowheads indicate pH3-expressing neurons with different immunolabeling intensity (black arrowhead: higher intensity; white arrowhead: lower intensity). (**B**, **C**) Quantitative analysis of pH3-labeling intensity in PrLCx (**B**) and ILCx (**C**). PrLCx: RHA Bs = 0.06 ± 0.004; RLA Bs = 0.06 ± 0.004; RHA FS = 0.12 ± 0.005; RLA FS = 0.10 ± 0.009; two-way ANOVA: (line) F_(1,18)_ = 4.93, p = 0.03^$^; (FS) F_(1,18)_ = 70.41, p < 0.0001***; (line x FS interaction) F_(1,18)_ = 3.48, p = 0.07; ILCx: RHA Bs = 0.07 ± 0.003; RLA Bs = 0.06 ± 0.003; RHA FS = 0.13 ± 0.003; RLA FS = 0.11 ± 0.002; two-way ANOVA: (line) F_(1,18)_ = 11.85, p < 0.003^$ $^; (FS): F_(1,18)_ = 154.81, p < 0.0001***; (line x FS interaction) F_(1,18)_ = 1.26, n.s. Bonferroni *post-hoc* test FS p < 0.05^§^. Student’s t-test for independent samples: p < 0.05^◊^). (**D-G**) Quantitative analysis of pH3-labeling intensity distributions in the PrLCx (**D**, **E**) and the ILCx (**F**, **G**) of each experimental group. PrLCx χ^2^ test: RHA Bs > RLA Bs, p < 0.05^#^; RHA FS > RLA FS, p < 0.001^###^; ILCx χ^2^ test: RHA Bs > RLA Bs, p < 0.001^###^; RHA FS > RLA FS, p < 0.01^##^). Number of animals in each experimental group: RHA Bs, n = 6; RLA Bs, n = 6; RHA FS, n = 5; RLA FS, n = 5. Scale bar = 20 μm.

### The phosphorylation of H3 induced by forced swimming in the PFCx may occur in the absence of concurrent ERK activation

To understand whether the activation of ERK may fully account for the phosphorylation of histone H3 [2], we analyzed the co-localization of pERK and pH3 in the PFCx under basal conditions and after FS (Fig 8A and 8D). Quantitative analyses revealed that under baseline conditions virtually every pERK-positive neuron in the PFCx of both Roman lines was also immunolabeled for pH3, with only a small percentage of neurons stained only for pERK (Fig 8B and 8E). On the other hand, ~ 50% of the pH3-positive neurons were also immunostained for pERK in both regions examined (Fig 8C and 8F). Interestingly, after FS there was a significant reduction in the percentage of neurons stained only for pERK in the PrLCx (Fig 8B). In contrast, FS increased the percentage of cells exclusively labeled for pH3 in both Roman lines (Fig 8C) in the same brain area. A different pattern of FS-induced changes in pERK and pH3 immunostaining was instead observed in the ILCx, where FS did not evoke any significant effect on the percentage of neurons immunostained only for pERK (Fig 8E), but increased the percentage of pH3-only positive neurons in both lines (Fig 8F). Taken together, these data suggest that the regulation of FS-induced H3 phosphorylation is, at least in part, mediated by signaling pathways independent from the ERK cascade.

**Fig 8:** The activation of ERK only partially overlaps with the expression of phosphorylated histone H3 in the PFCx. (**A**, **D**) Confocal micrographs showing double immunofluorescence for pERK (green) and pH3 (red) in the PrLCx (**A**) and in the ILCx (**D**). (**B**, **C**, **E** and **F**) Columns showing the mean percentage of cells labeled exclusively with pERK or pH3 compared to double positive cells in PrLCx (**B**, **C**) and ILCx (**E**, **F**) across experimental conditions in both Roman rat lines. PrLCx only pERK: RHA Bs = 8.4 ± 2.8%, RLA Bs = 10.8 ± 0.8%, RHA FS = 3.9 ± 2.4%, RLA FS = 0.00 ± 0%; two-way ANOVA: (line) F_(1,8)_ = 0.08, n.s.; (FS) F_(1,8)_ = 9.27, p < 0.03*; (line x FS interaction) F_(1,8)_ = 0.57, n.s.; only pH3: RHA Bs 44.2 ± 14.1%, RLA Bs = 61.2 ± 13.2%, RHA FS = 74.9 ± 5.2%, RLA FS = 76.1 ± 7.6%; two-way ANOVA: (line) F_(1,8)_ = 1.05, n.s.; (FS) F_(1,8)_ = 6.67, p < 0.05*; (line x FS interaction) F_(1,8)_ = 0.79, n.s.; ILCx only pERK: RHA Bs = 4.8 ± 2.9%, RLA Bs = 16.4 ± 0.1%, RHA FS = 15.3 ± 4.3%, RLA FS = 3.4 ± 2.5%; two-way ANOVA: (line) F_(1,8)_ = 0.00, n.s.; (FS) F_(1,8)_ = 0.08, n.s.; (line x FS interaction) F_(1,8)_ = 0.57, n.s.; only pH3: RHA Bs = 53.5 ± 12.7%, RLA Bs = 47.8 ± 7.6%, RHA FS = 68.7 ± 3.0%, RLA FS = 67.7 ± 3.0%; two-way ANOVA: (line) F_(1,8)_ = 0.27, n.s.; (FS) F_(1,8)_ = 7.36, p < 0.02*; (line x FS interaction) F_(1,8)_ = 0.14, n.s.). Number of animals in each experimental group: RHA Bs, n = 3; RLA Bs, n = 3; RHA FS, n = 3; RLA FS, n = 3. Scale bar = 50 μm.

## Discussion

RLA and RHA rats represent two divergent phenotypes respectively susceptible and resistant to display depression-like behavior in the forced swimming test, thereby providing a valid approach to investigate the neural circuitry and molecular mechanisms underlying stress-induced depression and to identify novel leads for the design of more efficacious therapies of depression in humans.

In the present study we show that an acute 15 min session of FS markedly increases the number of pERK- and pH3-expressing cells in various limbic brain areas of RHA and RLA rats with no statistically significant differences between the lines. However, the quantitative assessment of immunostaining intensities revealed that: (i) FS increases the mean levels of pERK and pH3 labelling in the PFCx of both Roman lines; (ii) under baseline and stressed conditions, neurons of the ILCx of RHA rats show higher levels of both pERK and pH3 immunostaining than their RLA counterparts; (iii) following FS, the levels of H3 phosphorylation are significantly higher in RHA vs. RLA rats also in neurons of the PrLCx; (iv) FS-induced phosphorylation of H3 in the PFCx may be mediated by signaling pathways independent from the ERK cascade.

The PFCx and the Acb play key roles in the control of the behavioral responses to aversive conditions [20]. Previous studies using brain microdialysis to assess dopamine release have shown that exposure to mild stressors, such as tail-pinch or the administration of anxiogenic drugs (i.e.: ZK-93426 and pentylenetetrazol), increases the functional tone of the mesocortical dopaminergic projections to the PFCx of RHA, but not RLA rats [20], whereas more robust or prolonged exposure to stressors affects dopamine release also in other dopaminergic terminal fields, such as the Acb ([29] and references therein). Notably, dopamine is able to increase ERK phosphorylation via stimulation of postsynaptic D1 dopamine receptors in several dopaminergic terminal fields. Thus, the increment in the extracellular concentration of dopamine in the PFCx and the Acb upon the inhibition of the presynaptic dopamine transporter by the systemic administration of cocaine [14,21] or MDMA (Ecstasy) is associated with an increase in the expression of pERK in the same brain areas, and this effect is prevented by the administration of a selective D1 dopamine receptor antagonist [22,30,31].

Therefore, based on the above findings, we predicted that (1) FS would increase the expression of pERK and pH3 in the PrLCx and ILCx as well as in the AcbCo and AcbSh of the Roman lines, and (2) the increment in the expression of pERK and, probably, of pH3 would be more robust in the PFCx of RHA *vs*. RLA rats because the increase in dopamine release induced by stressors in this brain area is more pronounced in the former than in the latter line [20].

Our results show that, in both Roman lines, FS elicits a robust increment in the number of pERK1/2-positive and pH3-positive cells in both subregions of the PFCx (i.e., PrLCx and ILCx) as well as a marked increase in the number of pERK1/2-positive cells in the AcbSh and AcbCo. To the best of our knowledge, this is the first report showing that FS is able to evoke the activation of ERK1/2 in the PFCx and Acb of the Roman rats, although this increment is quantitatively equivalent in both Roman lines for all the brain areas examined. Nevertheless, in keeping with our prediction, our data show that after FS the mean intensity of pH3 immunostaining is higher in the PrLCx and ILCx of RHA *vs*. RLA rats. Notably, the analysis of the frequency distribution of pH3 immunostaining intensity confirms the differences in the pH3 signal across lines both under basal conditions and after FS, as well as the larger number of cells showing high-intensity labelling for pERK in ILCx of RHA rats. Thus, these results are in line with our previous report showing that the functional tone of the mesocortical dopamine pathway is more robust in RHA rats as compared with their RLA counterparts [20]. Importantly, our study disclosed a plasticity-relevant pathway differentially regulated in the PFCx of these rat lines which is likely to reflect unique neuronal properties underlying their opposed responses to stressors. In this context, it will be interesting to assess whether the FS-induced increment in the intensity of pH3 immunostaining can be prevented by the administration of a selective D1 dopamine receptor antagonist.

Because the patterns of histone modifications, including H3 phosphorylation, correlate with global chromatin dynamics [2], our data suggest that changes in epigenetic regulation are likely to represent, or at least contribute to, the molecular mechanisms underlying the differential adaptive behavioral responses to stressful stimuli of RHA and RLA rats. Further studies are, therefore, warranted to identify the differences in posttranslational histone modifications and chromatin remodeling that distinguish the behavioral phenotypes of RHA and RLA rats.

The present study corroborates previous reports indicating that FS can evoke a robust increase in the expression of pERK1/2 in the Db, but not the Vb, of the DG [8]. This divergent responsiveness to stressful stimuli may be explained by morphological and functional differences between the transverse axis of the DG. In this context, it has been suggested that anatomical differences between Vb and Db may account for their specific contribution to learning and memory formation [32]. In support of this suggestion, Barnes et al. have described an asymmetry in the activation of immediate-early genes along the axis of the DG. Thus, exploratory behavior is associated with an increase in the density of Arc-expressing cells exclusively in the dorsal blade [33].

Notably, at variance with Gutiérrez-Mecinas et al. [8], who reported that acute stress-evoked ERK phosphorylation is restricted to the DG, we found that the expression of pERK is markedly increased by FS not only in the DG, but also in the PFCx, as well as in the Acb of RHA and RLA rats. In agreement with our data, Shen and colleagues reported an increase of pERK 2 in the neocortex, the PFCx, and the striatum upon FS [10]. It is unlikely that the above mentioned contrasting results are due to strain-related factors, since Gutiérrez-Mecinas et al. carried out their experiments in Wistar rats, the strain from which the Roman lines derive.

It has been shown that the glucocorticoid hormones released as a part of the stress response evoked by FS can bind to and activate their specific receptors located in the granule neurons of the DG, thereby inducing a rapid enhancement of ERK phosphorylation [7,8]. The pERK1/2-mediated activation of target kinases such as MSK1 and Elk-1 [34] leads to the phosphorylation and acetylation of histone H3, thereby inducing c-Fos and Egr-1 expression [8]. These chromatin remodeling mechanisms evoked by FS, which take place in the granule neurons of the DG, are involved in the encoding of memories of stressful events [26]. It is noteworthy that these effects are mediated by the activation of both, glucocorticoid and N-methyl-D-aspartate (NMDA) receptors, as indicated by the finding that they are completely blocked by the systemic administration of the glucocorticoid receptor antagonist mifepristone and the NMDA receptor antagonist dizocilpine [8]. Importantly, there is growing evidence supporting a dysregulation of the HPA axis in the RLA line; thus, the activation of the HPA axis induced by mild stressors is more robust in RLA than RHA rats and, under dexamethasone suppression, RLA rats exhibit a more pronounced response to CRH than their RHA counterparts [35]. On the basis of the above findings, it was expected that FS would induce a more robust increment in pERK expression in the DG of RLA *vs*. RHA rats. Conversely, we found that FS increases to the same extent the expression of pERK1/2 in the Db of the DG of both Roman lines. This result could be explained by the involvement of other signaling cascades activated by a psychological stressor such as the aforementioned NMDA glutamate receptors [2]. Thus, a plausible explanation for our results is that a more robust stress-induced activation of the HPA axis in RLA *vs*. RHA rats may be compensated by a less intense activation of the NMDA receptor-mediated glutamatergic neurotransmission in RLA rats as compared with their RHA counterparts. Further experiments are therefore required to test this hypothesis.

To investigate whether the activation of pERK1/2 produced by FS is instrumental for the phosphorylation of histone H3, we used double immunofluorescence and confocal microscopy to evaluate the percentage of pERK and pH3 co-localization in neurons of the PrLCx and the ILCx. We found that, under basal conditions, almost the entirety of pERK-expressing neurons in both areas of RHA and RLA rats is also pH3-positive. In contrast, about one half of the pH3-positive cells does not show pERK immunolabelling. Interestingly, following FS, the percentage of neurons expressing exclusively pERK in the PFCx decreases, while the percentage of neurons stained only for pH3 is significantly increased. In addition, the phosphorylation of H3 elicited by FS in the PFCx takes place mainly in neurons that do not express pERK suggesting that such H3 modification is mediated by a different intracellular signaling pathway. In support of an uncoupling between the ERK1/2 pathway and H3 phosphorylation, we previously reported that H3 phosphorylation induced by morphine-withdrawal in Wistar rats is only partially linked to ERK activation depending on the specific brain region [4]. Although it cannot be ruled out that the increase in H3 phosphorylation results from an early and short lived wave of ERK activation, which would not be detected under our experimental conditions, this is an unlikely possibility. Indeed, based on previous observations of our and other groups [4,36,37], the time course to detect full ERK activation seems totally compatible with the experimental protocol employed in the present study (15 min after stimulation). Additional experiments are therefore warranted to explore alternative signaling cascades that may lead to H3 phosphorylation such as the CaMKII pathway.

In conclusion, we showed that the increment in the number of pERK 1/2- and pH3-expressing cells evoked by FS is not restricted to the Db of the DG as previously reported [8], but is also observed in the PFCx and Acb of RHA and RLA rats; moreover, nerve cells located in the PFCx of RHA rats show higher rates of pH3 and pERK than those of the RLA line. Such variations in the intracellular signaling cascades may be involved in the different coping strategies displayed by the Roman lines in the face of stressful conditions.
